# Adrenal Disorders and the Paediatric Brain: Pathophysiological Considerations and Clinical Implications

**DOI:** 10.1155/2014/282489

**Published:** 2014-09-03

**Authors:** Vincenzo Salpietro, Agata Polizzi, Gabriella Di Rosa, Anna Claudia Romeo, Valeria Dipasquale, Paolo Morabito, Valeria Chirico, Teresa Arrigo, Martino Ruggieri

**Affiliations:** ^1^Department of Pediatric Neurology, Chelsea and Westminster Hospital NHS Foundation Trust, 369 Fulham Road, London SW10 9NH, UK; ^2^Unit of Genetics and Paediatric Immunology, Department of Pediatrics, University of Messina, Italy; ^3^National Center for Rare Diseases, Istituto Superiore di Sanità, Rome, Italy; ^4^Institute of Neurological Sciences, National Research Council, Catania, Italy; ^5^Infantile Neuropsychiatry Unit, Department of Pediatrics, University of Messina, Italy; ^6^Department of Clinical and Experimental Medicine and Pharmacology, University of Messina, Italy; ^7^Chair of Pediatrics, Department of Educational Sciences, University of Catania, Italy

## Abstract

Various neurological and psychiatric manifestations have been recorded in children with adrenal disorders. Based on literature review and on personal case-studies and case-series we focused on the pathophysiological and clinical implications of glucocorticoid-related, mineralcorticoid-related, and catecholamine-related paediatric nervous system involvement. Childhood *Cushing syndrome* can be associated with long-lasting cognitive deficits and abnormal behaviour, even after resolution of the hypercortisolism. Exposure to excessive *replacement of exogenous glucocorticoids* in the paediatric age group (e.g., during treatments for adrenal insufficiency) has been reported with neurological and magnetic resonance imaging (MRI) abnormalities (e.g., delayed myelination and brain atrophy) due to potential corticosteroid-related myelin damage in the developing brain and the possible impairment of limbic system ontogenesis. *Idiopathic intracranial hypertension* (IIH), a disorder of unclear pathophysiology characterised by increased cerebrospinal fluid (CSF) pressure, has been described in children with hypercortisolism, adrenal insufficiency, and hyperaldosteronism, reflecting the potential underlying involvement of the adrenal-brain axis in the regulation of CSF pressure homeostasis. Arterial hypertension caused by *paediatric adenomas* or *tumours* of the *adrenal cortex* or *medulla* has been associated with various hypertension-related neurological manifestations. The development and maturation of the central nervous system (CNS) through childhood is tightly regulated by intrinsic, paracrine, endocrine, and external modulators, and perturbations in any of these factors, including those related to *adrenal hormone imbalance*, could result in consequences that affect the structure and function of the paediatric brain. Animal experiments and clinical studies demonstrated that the developing (i.e., paediatric) CNS seems to be particularly vulnerable to alterations induced by adrenal disorders and/or supraphysiological doses of corticosteroids. Physicians should be aware of potential neurological manifestations in children with adrenal dysfunction to achieve better prevention and timely diagnosis and treatment of these disorders. Further studies are needed to explore the potential neurological, cognitive, and psychiatric long-term consequences of high doses of prolonged corticosteroid administration in childhood.

## 1. Background

The assumption that children respond similarly to adults with respect to disease pathophysiology, medication efficacy, and adverse reactions is often erroneous [1].

It is largely known that the developing central nervous system (CNS) is qualitatively different from the adult nervous system, as the latter represents the final result of a complex ontogenetic process that requires various steps of cellular proliferation, angiogenesis, migration, synaptogenesis, differentiation, and myelination [2]. Evidence from numerous sources has demonstrated that neural development processes extends from the embryonic period through adolescence [2, 3].

The development of the nervous system is sensitive to potential insults during vulnerable periods because the process is dependent on the temporal and regional emergence of critical developmental processes (i.e., proliferation, migration, differentiation, synaptogenesis, myelination, and apoptosis) [3].

The ontogeny of the CNS in childhood is under tight regulation by intrinsic, paracrine, endocrine, and external modulators, and perturbations in any of these factors could result in long-term consequences that possibly lead to long-term impairment of the structure and function of the developing brain [3, 4].

In this context, among the modulator substances, adrenal hormones exert very important regulatory activities and trophic effects on cell survival, differentiation, maturation, and synaptogenesis of the CNS [5].

Adrenal hormones are secreted by the adrenal glands, which contain three zones within the cortex (i.e., glomerulosa, fasciculate, and reticularis), whereas the adrenal medulla is located in the central portion of the gland. The adrenal cortex is derived from the mesoderm, while the adrenal medulla is derived from the neuroectoderm, and its chromaffin cells secrete catecholamines in a process regulated by the preganglionic sympathetic neurons. The zona reticularis adjacent to the medulla secretes sex hormones, and the middle zone (i.e., fasciculate) secretes glucocorticoids (e.g., cortisol); the secretion from both of these zones is under the control of the hypothalamus-pituitary axis. The outer zone (i.e., glomerulosa) secretes mineralocorticoids (e.g., aldosterone) and is under the control of the renin-angiotensin system (RAS) [6].

A wide array of conditions can cause adrenal disorders in the paediatric age group, with a higher percentage of underlying causative genetic diseases compared to the adult age group. Despite extensive evidence from animal experiments regarding the higher risk of corticosteroid-related neurological sequelae in the developing brain, a limited number of human studies have functionally investigated the impact of adrenal disorders on the paediatric brain and have fully longitudinally explored the potential neurological and psychiatric long-term consequences of both endogenous and exogenous adrenal hormone imbalances.

In this paper, we discuss the most frequent paediatric adrenal disorders, with an emphasis on their neurologic manifestations, their pathophysiology, and their diagnosis.

## 2. Hypercortisolism and the Paediatric Brain

Cushing syndrome is a metabolic disorder caused by chronically high levels of endogenous cortisol or by exogenous exposure to corticosteroids that impairs carbohydrate, protein, and lipid metabolism and includes all causes of hypercortisolism; on the other hand, the term Cushing disease is reserved for cases of pituitary-dependent Cushing syndrome. The overall incidence of Cushing syndrome is approximately 2 to 5 new cases per million people per year, and only approximately 10% of the new cases each year occur in children [7]. A common cause of Cushing syndrome in children is chronic glucocorticoid administration. Cushing disease (i.e., pituitary dependent) accounts for approximately 75% of all cases of Cushing syndrome in children older than 7 years. In children under 7 years, Cushing disease is less frequent, and the adrenal causes of Cushing syndrome (i.e., adenoma, carcinoma, or bilateral hyperplasia) represent the most common causes of the condition in infants [8]. Adrenal cortical neoplasms in paediatric patients are more difficult to diagnose, and it is also more difficult to separate benign from malignant tumours in this age group [9, 10].

Ectopic corticotropin (ACTH) production accounts for less than 1% of the cases of Cushing syndrome in adolescents, and it is very rare in younger children [8].

Primary pigmented adrenocortical nodular disease (PPNAD; MIM 610489) is a dominantly inherited genetic disorder with the majority of cases associated with Carney Complex type 1 (CNC1; MIM 160980). CNC1 complex is a multiple endocrine neoplasia (MEN) syndrome that affects endocrine glands such as the adrenal cortex (causing Cushing's syndrome), the pituitary, and the thyroid. PPNAD is associated with germ line inactivating mutations of the PRKAR1A gene, which is located at 17q22-24 and encodes protein kinase A [10].

Bilateral adrenocortical hyperplasia has also been reported in McCune-Albright syndrome (MAS; MIM 174800), but in these cases, it is not always associated with hypercortisolism. In MAS, there is a somatic mutation of the GNAS1 gene leading to constitutive activation of the Gsα protein and non-ACTH-dependent adrenal cortex steroidogenesis [7, 9].

The onset of Cushing syndrome in children is often subclinical and insidious, with the most common presenting symptom being weight gain in the absence of a concomitant height gain [7, 8]. This abnormal growth can be associated with various other clinical signs and symptoms including facial plethora (see Figure 1), hypertension, amenorrhea, and skin manifestations such as acne, easy bruising, striae rubrae, and acanthosis nigricans [7–9]. Hyperandrogenism is another frequent feature of Cushing syndrome, which is due to the increase of adrenal androgens related to ACTH or to their autonomous production by adrenal tumors. Signs and symptoms include* acne*, scalp hair loss (*androgenic alopecia*), and excessive facial and body hair (*hirsutism*) [8, 9].

Of note, adults with Cushing syndrome frequently have cognitive impairment and psychiatric disturbances (mainly depression and anxiety) with a ratio between 57% and 79% [11, 12], while children with this disorder show rates of psychiatric symptoms of 44%, with compulsive behaviours predominating [13].

Also exogenous corticosteroid administration has been often reported to be associated with psychiatric manifestations, including psychotic symptoms, hyperactivity, and mild changes in mood and cognition; these manifestations can appear during corticosteroid treatment or during withdrawal [14]. Although the pathophysiology of these side effects is still not fully understood, some authors have proposed potential glucocorticoid-related hippocampus damage as the cause [15]. Concerns have been raised regarding the potential for hippocampus damage that is not completely reversible in some children treated with corticosteroids (especially those on the highest doses and long-term therapies), with possible long-lasting negative effects on cognition, but no longitudinal studies have been performed to clarify the cognitive outcomes in these patients [16].

Of note, several studies have reported a significant global loss of brain volume and CNS atrophic changes based on radiological investigations of both adult and paediatric patients with Cushing Syndrome [17–19]. In addition, supraphysiological doses of exogenous glucocorticoids were found to possibly cause cerebral atrophy and volume loss in different paediatric series [20, 21], and other studies demonstrated a possible link between the increased activity of the pituitary-adrenal axis and cerebral atrophy in the context of depression and stress [22].

In most patients, the MRI atrophic changes related to hypercortisolism are detected in the amygdala, temporal lobe, and hippocampus [17–19, 21], and this could explain the behavioural abnormalities and the impairment of cognition and memory, given the high biological importance of these brain regions in the processing of emotions and in cognition.

Of note, significant recovery of depressive symptoms and improvement in cognition and reversal of cerebral atrophy have been observed in adult patients with Cushing syndrome after clinical remission [17].

Data on the evolution of the cerebral atrophy following correction of hypercortisolism are limited in the paediatric age group, but in a study of 11 children with Cushing syndrome followed up after surgery, a long-lasting significant decline in cognitive function was observed after a return to eucortisolism, despite almost complete reversal of the cerebral atrophy [19]. This observation is in contrast to the adult experience, and the possible decline in cognitive function after curing Cushing syndrome seems to be unique to the paediatric population.

### 2.1. Pathophysiology of Glucocorticoid-Related Paediatric Brain Damage

The pathogenesis of the loss of brain volume induced by chronic glucocorticoid excess appears to be multifactorial and is not yet fully understood.

Glucocorticoids can act both on mineralcorticoid receptors (MRs) and on glucocorticoid receptors (GRs). MRs are usually protected by glucocorticoids exposure by the effects of 11*β*-HSD2 enzyme, which converts cortisol into the inactive cortisone; however, 11*β*-HSD2 is not expressed in the hippocampus or other limbic structures, allowing MRs activation by glucocorticoids in these latter brain regions [23]. Therefore, glucocorticoids excess increases the occupation of MRs/GRs, with predominant involvement of some (but not other) brain regions (e.g., limbic system).

Notably, studies on hippocampal cell cultures showed that supraphysiological doses of glucocorticoids lead to a reversible phase of atrophy of the apical dendrites of pyramidal neurons [24]. In addition, glucocorticoids have been shown to increase the synaptic accumulation of glutamate and to stimulate the N-methyl-D-aspartate (NDMA) receptors with a subsequent increase in intracellular cytosolic Ca^+^ in postsynaptic neurons, which activate several processes leading to neuron cell death [19, 22].

Of note, the partial reversibility of brain atrophy after a return to eucortisolism would indicate that the above-discussed MRI abnormalities are not exclusively related to neuronal death. Interestingly, among the exogenous corticosteroids, dexamethasone has been classically regarded as very potent in treating cerebral oedema [25]; therefore, the loss of brain volume in Cushing syndrome could be putatively secondary also to a decrease in water content of the brain due the hypercortisolism [26].

Interestingly, the complications related to exogenous and endogenous corticosteroid excess on the paediatric brain might depend on several variables, including the stage of CNS development at the time of exposure and the duration of exposure, and in the case of exogenous compounds, the pharmacological characteristics of the corticosteroids used and their dosage [5].

A very important variable might be represented by the stage of CNS development at the time of exposure. In this regard, the neurological manifestations could to be directly proportional to the immaturity of the brain, and the foetal age appears as the most “at risk” period of life [5, 27]. In fact, there is considerable evidence from animal models (e.g., baboon and sheep) that antenatal administration of steroids can have detrimental effects on the developing CNS, causing a dose-dependent brain atrophy (e.g., predominantly in the hippocampus) and delay in myelination [27, 28].

Notably, the prenatal administration of corticosteroids in humans is common clinical practice in women with possible preterm delivery and is used to stimulate lung maturation and prevent respiratory distress syndrome. The neurological outcomes of those treated infants are still a matter of debate. In fact, several long-term clinical studies have shown no impact of antenatal corticosteroid therapy on neurodevelopmental outcomes during the follow-up of these children (e.g., at 2 years of age) [29–31]. Conversely, other studies suggest a higher rate of cerebral palsy in infants exposed to repeat courses of corticosteroids [32], as well as neurodevelopmental abnormalities [33] and behavioural effects [34].

These observations suggest that prolonged exposure to excess glucocorticoids from an endogenous or exogenous source, not only significantly impacts the weight, height, and development of children, but may also have permanent effects on the paediatric developing brain, behavior, and cognition.

## 3. Adrenal Insufficiency and the Paediatric Brain

Primary adrenal insufficiency, or Addison's disease, is the destruction or dysfunction of the adrenal cortex gland causing impaired secretion of glucocorticoids and mineralocorticoids [35, 36]. Adrenal insufficiency is a rare disorder with a prevalence in developed countries of up to 93–144 cases per million, with an estimated incidence of 4.44–6 new cases per million population per year [36, 37]. In developed countries, has been estimated that 80–90% of cases of primary adrenal insufficiency are caused by the destruction of the adrenal cortex by cell-mediated immune mechanisms, which can be isolated (40%) or part of an autoimmune polyendocrinopathy syndrome (60%) [36].

Of note, in the paediatric age group, adrenal insufficiency is in most cases related to genetic disorders including impaired steroidogenesis due to defects in enzymes involved in hormone production (e.g., congenital adrenal hyperplasia) or developmental defects of the glands, often associated with mental retardation and neurological features (e.g., Smith-Lemli-Opitz syndrome, triple A syndrome) [11, 36].

In a large series of 103 children with Addison's disease, most reported causes were genetic conditions, which accounted for 78% of cases, whereas autoimmune disease was diagnosed in only 13% of cases [38]. Secondary adrenal insufficiency results from pituitary disease that hampers the release of ACTH exclusively impairing glucocorticoid secretion; tertiary adrenal insufficiency is in most cases related to the long-term administration of exogenous glucocorticoids, which leads to prolonged suppression of hypothalamic secretion of CRH [35, 36].

Adrenal insufficiency in children typically presents with insidious nonspecific symptoms such as fatigue, malaise abdominal pain, weight loss, nausea, and vomiting. Physical signs appear as later manifestations of the disease and include hypotension and hyperpigmentation (e.g., in the primary forms). Classic biochemical signs include hyponatremia, hyperkalaemia, hypoglycaemia, and ketonaemia [36, 37]. A life-threatening adrenal crisis can be the first presentation of adrenal insufficiency, with sudden onset of vomiting, abdominal pain, myalgia, severe hypotension, and hypovolaemic shock. This acute presentation is usually precipitated by a physiological stress, such as surgery, trauma, or a concurrent infection.

In some paediatric reports, adrenal insufficiency has been reported in association also with idiopathic intracranial hypertension (IIH; see Section 4.2), with neurological symptoms (e.g., headache, diplopia) that appeared as the first clinical manifestations, before those related to the adrenal insufficiency [39, 40].

There have been a number of studies or single case descriptions reporting on isolated episodes of hypoglycaemic coma and on multiple cases of extrapontine and central pontine myelinolysis with encephalopathy and coma in children with Addison disease [41–43]. Adrenal insufficiency is often associated with chronic severe hyponatraemia. Rapid correction of chronic hyponatremia leads to a significant brain dehydration as potassium and organic substances cannot be introduced into the cells as fast as required [44]. As a result of that, the myelin sheath is stripped from the axon and the oligodendrocytes are damaged, especially in some brain areas, which are more vulnerable to the osmotic damage (e.g., pons, basal ganglia), with consequent regional-limited demyelination [45].

Therefore, both extra pontine and central pontine myelinolysis can occur as a consequence of a rapid correction of hyponatremia in individuals with chronic, severe hyponatraemia [45]. The initial symptoms of pontine myelinolysis, which manifest shortly after the rapid correction of hyponatremia, include a depressed level of awareness, difficulty in speaking (dysarthria or mutism), and difficulty in swallowing (dysphagia). Seizures, global tremor and a wide array of movement disorders can be also present at onset, especially when are involved the extra pontine regions (e.g., basal ganglia). Additional symptoms often arise over the following 1-2 weeks including loss of consciousness, global weakness, paralysis in the arms and/or the legs, stiffness, and difficulty with coordination [46]. Myelinolysis can be reversible or, in the most severe cases, can also lead to coma and death. In patients with chronic hyponatremia (e.g., in adrenal insufficiency), the rate of correction should be less than 0.5 mmol/L/h to prevent central and extra pontine myelinolysis [47, 48].

### 3.1. Congenital Adrenal Hyperplasia

In the paediatric age group, the most common cause of primary adrenal insufficiency is* congenital adrenal hyperplasia* (CAH), a complex and heterogeneous condition resulting from a genetic defect in the biosynthetic pathway of cortisol and/or aldosterone in the adrenal cortex.

In a large series of 103 children with Addison's disease, CAH was revealed as the most frequent cause of adrenal insufficiency, accounting for 71.8% of the cases [38]. Classic CAH is an autosomal recessive disorder with a prevalence rate estimated at one in 15,000 live births [53].

The most common form is classic CAH due to* 21-hydroxylase* deficiency (MIM 202010), a condition characterised by low synthesis of glucocorticoids and, in many cases, mineralocorticoids (i.e., in the salt loosing variant) and adrenal hyperandrogenism. More rare forms are caused by deficiency of* 11*β*-hydroxylase*,* 17α-hydroxylase*,* 3*β*-hydroxysteroid dehydrogenase*, or* P450 oxidoreductase* [53].

Replacement of glucocorticoids is necessary for patients with CAH; treatment with mineralocorticoids is necessary in these patients only when aldosterone production is deficient (e.g., in the salt loosing variant). Since intrauterine life, prenatal glucocorticoid deficiency has a potential impact on the foetal brain, and as evidence of this, a significant decrease in the amygdala volume has been observed in CAH infants, suggesting a prenatal critical effect of hormone deficiency on the developing CNS [54].

Of note, several studies based on MRI have described brain white matter abnormalities in children with CAH, with the radiological changes that can be sometimes detected from the first days of life in children with classic CAH [49, 55]. In addition to the white matter changes, moderate atrophy in the right temporal cortex, small volume hippocampus, and agenesis or thinning of the corpus callosum were observed in the long term follow-up of children with classic CAH [56–58].

The pathophysiology of white matter abnormalities is still not fully understood, but many authors have proposed that exposure to excess exogenous glucocorticoids during CAH treatment is the most feasible explanation for these MRI findings due the potential inhibitory role of cortisol in the process of neuronal maturation and myelination by inhibiting the differentiation of oligodendrocyte precursors [5, 28, 56, 57]. In addition, hyponatremia, potentially leading to myelinolysis, has been suggested as a potential contributing factor to the impaired myelin formation in these patients [55, 56]. Some authors have also suggested that hormonal imbalance related to a deficiency in cortisol and aldosterone and an overproduction of 17-OH-progesterone and androgen may further cause a destabilisation of the myelin molecule leading to its degeneration [56].

Clinically, these children may present with seizures, lethargy, postural and intentional tremor, tendon reflex asymmetry, or cerebellar symptoms [49, 55–58]. Standard MRI sequences performed in the first days of life in some newborns with classical CAH typically showed diffuse hyperintensity on T1-weighted sequences (Figure 2(a)), with reduced diffusion in the periventricular white matter on the diffusion-weighted imaging (DWI) sequences. Follow-up radiological studies often showed complete reduction in the previously detected imaging abnormalities (Figure 2(b)), although long-lasting abnormalities and irreversible atrophic changes have also been documented in some patients [55].

Neurological outcomes have not been systematically reported in these children, but a mild reduction in cognitive capacities and memory has been described in some, likely due to the effects of supraphysiological doses of corticosteroid replacement on the amygdala and hippocampus development [59, 60].

### 3.2. X-Linked Adrenoleukodystrophy

*X-linked adrenoleukodystrophy* (X-ALD; MIM 300100) is the most common peroxisomal disorder, with an estimated birth incidence of 1 in 17,000 newborns (male and female) [61]. It is caused by mutations in the* ABCD1* gene located on the X-chromosome that encodes the peroxisomal membrane protein ALDP, which is involved in the transmembrane transport of very long-chain fatty acids (VLCFA); therefore, a defect in ALDP results in elevated levels of VLCFA in the plasma and tissues [62].

Adrenoleukodystrophy has a variable age of onset in childhood and exhibits different phenotypes. The clinical spectrum in males with X-ALD ranges from isolated adrenocortical insufficiency and slowly progressive myelopathy to devastating diffuse cerebral demyelination.

X-ALD is a frequent cause of Addison's disease in boys and adult males. Adrenal insufficiency (or even Addisonian crisis) can sometimes be the presenting symptom of X-ALD in boys and men, years or even decades before the onset of neurological symptoms [10, 36, 62]. The most aggressive and devastating phenotype is cerebral ALD, consisting of a rapidly progressive demyelinating condition that affects the cerebral white matter. It is by definition confined to boys who develop cerebral involvement before the age of 10 years. The boys are normal at birth and have unremarkable development. The mean age of onset is approximately 7 years [62].

The disease usually manifests early with behavioural manifestations including inattention and hyperactivity. It often becomes apparent through school difficulties. It progresses to visual symptoms, auditory processing difficulties, and motor incoordination. Later neurological manifestations can include moderate dystonia, pyramidal signs, gait disturbances with features of cerebellar and pyramidal tract involvement, hemiparesis, or spastic tetraparesis [10, 61, 62]. Typical MRI white matter changes include signal hyper intensities on T2-weighed and FLAIR sequences in the parietooccipital region and the splenium of the corpus callosum [61, 62].

Although it is still impossible to predict which patients will develop the neurological manifestations of the disease, it has been estimated that approximately 35–40% of children with mutations in the ABCD1 gene will develop cerebral ALD before adulthood [61, 62].

However, the prognosis is variable with a great variability between the patients and depends on the neuroinflammatory stage of the disease, which correlates with the cerebral demyelination and the neurological manifestations. It is likely that if they survive into adulthood, all patients with X-ALD eventually develop adrenomyeloneuropathy (AMN), a condition characterised by paraparesis, spasticity, and signs of neuropathy, with onset usually after 20 years of age [10, 63].

The only treatment that has shown some clear benefits in early symptomatic X-ALD is based on haematopoietic stem cell transplantation (HST), with stabilisation or improvement in the clinical and/or MRI findings in 50–75% of treated boys [64]. In the future, HST with autologous cells that have been genetically corrected with lentiviral vectors and reinfused might become an effective treatment because of the promising preliminary results [65].

Paediatric endocrinologists and neurologists may face X-ALD and should potentially consider this disease in any boy presenting with Addison's disease. Early recognition of X-ALD is very important because in some cases, treatment is available, such as HCT in the early stages of cerebral ALD and endocrine replacement therapy for adrenal insufficiency.

### 3.3. Other Genetic Forms of Adrenal Insufficiency

*Autoimmune polyglandular syndrome type 1* (APS-1; MIM 240300) is a rare autosomal recessive disorder caused by mutations in the autoimmune regulator (AIRE) gene, that is characterised by autoimmune adrenal insufficiency, hypoparathyroidism, chronic mucocutaneous candidiasis, ectodermal dystrophy, and many other potential autoimmune disorders. Children with APS-1 may have autoimmune activation against CNS antigens such as autoantibodies directed against aromatic L-amino acid decarboxylase (AADC), tyrosine hydroxylase (TH), tryptophan hydroxylase (TPH), and glutamic acid decarboxylase (GAD). Neurological symptoms previously described in association with APECED include the stiff-man syndrome, cerebellar ataxia, inflammatory demyelinating polyneuropathy, and acute reversible CNS demyelination [66, 67].

*Congenital adrenal hypoplasia* (MIM 300200), due to* complex glycerol kinase* deficiency, is an X-linked condition in which the adrenal cortex development is prevented. In this disorder, the onset of symptoms varies from birth to childhood, and the clinical presentation includes adrenal insufficiency, psychomotor retardation, muscular dystrophy, hypertelorism, strabismus, short stature, and osteoporosis [68].

*Triple A syndrome *(MIM 231550) is an autosomal recessive disorder that consists of the triad of ACTH-resistance adrenal insufficiency, alacrima, and achalasia. Aldosterone deficiency may also be observed in patients with gradual neurologic dysfunction with polyneuropathy, mental retardation, hyperreflexia, muscle weakness, dysarthria, ataxia, and abnormal autonomic function [69, 70].

*Smith-Lemli-Opitz syndrome* (SLOS; MIM 270400) is a neurodevelopmental disorder caused by inborn errors of cholesterol metabolism resulting from mutations in 7-dehydrocholesterol reductase (DHCR7) characterised by intellectual disability, CNS malformations (e.g., abnormalities in septum pellucidum and in corpus callosum, colpocephaly, arachnoid cysts, type I Chiari malformation), and multiple congenital anomalies and is possibly associated with adrenal insufficiency due to the impaired steroidogenesis [36, 37].

*Kearns-Sayre syndrome *(KSS; MIM 530000) is a mitochondrial disease characterised by myopathy, ptosis, ophthalmoplegia, and deafness and can also manifest with endocrine anomalies, including adrenal insufficiency [10, 36].

## 4. Hyperaldosteronism and the Paediatric Brain

Hyperaldosteronism is a condition characterised by an increase in mineralocorticoid secretion due a disorder of the zona glomerulosa of the adrenal glands [71].

Primary hyperaldosteronism (PAL) is an exceptional entity in the paediatric age group and is caused by aldosterone secreting adenomas (or carcinomas), bilateral adrenal hyperplasia (e.g., idiopathic hyperaldosteronism), or primary unilateral adrenal hyperplasia [71, 72]. The renin activity is typically low in all forms of PAL because of the negative feedback effect.

Familial hyperaldosteronism (FH) is a rare autosomal dominant disorder with two main typical presentations (i.e., types 1 and 2). The FH type 1 (MIM 103900) is characterised by hypertension, weakness, failure to thrive, and increased incidence of intracranial aneurysms [73]. Typical laboratory features are hyperaldosteronism and high levels of hybrid steroids (e.g., 18-hydroxycortisol and 18-oxocortisol); excellent clinical response to exogenous glucocorticoid administration has been achieved. The FH type 2 (MIM 605635) is characterised by aldosterone-producing adenomas or bilateral idiopathic hyperaldosteronism (or both), and it usually does not respond to glucocorticoids [73].

Secondary hyperaldosteronism (SAL) results from overactivation of the renin-angiotensin system (RAS) and is therefore characterised by elevated aldosterone and renin levels and usually occurs in adults with renovascular hypertension or renin-secreting tumours. The most frequent causes of SAL in the paediatric age group are the salt-losing tubulopathies (e.g., Bartter syndrome, Gitelman syndrome), autosomal recessive conditions characterised by the loss of Na^+^ from the distal nephron with consequent RAS activation and persistent SAL. These disorders variably manifest with growth failure, hypokalaemia, metabolic alkalosis, hyperreninaemia due the hyperplasia of the juxtaglomerular apparatus, and hyperaldosteronism; the arterial pressure is usually within normal limits [72, 74].

Other causes of hyperaldosteronism include potassium sodium-wasting nephropathy, renal tubular acidosis, diuretic or laxative abuse, nephrotic syndrome, nephropathic cystinosis, oestrogen administration, and recombinant growth hormone (r-GH) treatment [75].

Hyperaldosteronism (and the consequent activation of MRs pathways that are present in different organs and tissues including kidney and brain) is one of the most important causes of endocrine-related arterial hypertension, potentially leading to neurological complications as stroke and hypertensive encephalopathy (see Sections 4.1 and 5) [76]. Additionally, hyperaldosteronism has been recently regarded as a cause of IIH, due to a potential impairment of cerebrospinal fluid homeostasis in the presence of an underlying MRs overactivation in the choroid plexus epithelium (see Section 4.2) [77].

### 4.1. Pseudohyperaldosteronism and Pseudohypoaldosteronism and the Paediatric Brain

Congenital absence of adrenal enzymes such as* 11*β*-hydroxylase *and* 17α-hydroxylase* lead to CAH with elevated serum deoxycorticosterone (DOC). Supraphysiological levels of DOC promote salt retention, volume expansion, and arterial hypertension, similarly to what occur in hyperaldosteronism [75].

Apparent mineralcorticoid excess (AME; MIM 218030) is caused by deficiency of* 11*β*-hydroxysteroid dehydrogenase type 2* (11*β*HSD2). This condition is characterised by decreased conversion of biologically active cortisol into inactive cortisone, with consequent constitutional MRs activation, resulting in pseudohyperaldosteronism and suppressed levels of both renin and aldosterone [78].

AME has been frequently reported in association with neurological manifestations in the pediatric population. In a series of 14 children with AME, 8 had neurologic symptoms at the time of diagnosis including developmental delay, abnormal electroencephalographic evaluation with a pattern of generalized seizure disorder, history of lapses of awareness and signs of cerebral infarcts on MRI [79]. Notably, stroke represents one of the most dangerous risk factors for children with AME, possibly due the detrimental effects on the cerebral vessels of constitutive activation of the MRs, largely expressed in many CNS sites [80]. In a report, a female adolescent with AME developed stroke despite adequate treatment of her hypertension and the authors suggested a pathophysiological role of 11*β*HSD2 deficiency as causative factor of endothelial dysfunction involving the cerebral circulation, due to the excessive exposure to high levels of circulating active cortisol [81].

Pseudohypoaldosteronism (PHA) is a condition characterised by mineralocorticoid resistance, with a great genetic and clinical heterogeneity [82]. PHA type 1 can result from autosomal dominant mutations in the mineralocorticoid receptor coding gene NR3C2 (PHA1A; MIM 177735) or from autosomal recessive mutations in the epithelial sodium channel (PHA1B; MIM 264350). Both autosomal dominant and recessive forms of PHA1 are characterised by salt wasting and hyperkalaemia with increased plasma renin and aldosterone levels, reflecting a resistance of the kidney and other tissues to mineralocorticoids [83]. The onset of clinical manifestations in PHA1 is mainly confined to early childhood, with hyperkalaemia, hyponatremia, and dehydration. Salt supplements are required (especially in the recessive form that is more severe) coupled with attainment of control of hyperkalaemia [83]. PHA1 has been described in association with encephalopathy and convulsions, due to rapid (erroneous) salt supplementation and possible underlying pontine and/or extrapontine myelinolysis [84].

PHA type 2 (PHA2) represents a group of conditions commonly characterised by hyperkalaemia despite normal renal glomerular filtration, metabolic acidosis, and a low plasma renin level, with high incidence of hypertension. Plasma aldosterone levels are low to mildly (but inadequately) increased. PHA2 is characterised by a great genetic variability with several potentially causative genes (including* WNK1*,* WNK4*,* KLHL3*, and* CUL3*), most of them crucially involved in the (negative) regulation of the NaCl cotransporter (NCC) [85, 86].

In PHA2, recurrent myalgia and periodic paralysis had been recorded in the original description by Gordon [87]. Mutations in the* WNK1* gene have been shown to be causative of the hereditary sensory neuropathy in a French family with PHA2 and defects in peripheral sensory perception; the authors demonstrated that WNK1* is highly *expressed in the sensory components of peripheral nervous system and is associated with relaying sensory and nociceptive signals in sensory neurons [86, 88].

### 4.2. Hyperaldosteronism and IIH

IIH, also known as* pseudotumor cerebri*, is a neurological disorder of uncertain aetiology, characterised by increased intracranial pressure (ICP) in the absence of a tumour, hydrocephalus and no apparent cause based on neuroimaging or other routine evaluations [89]. Its main symptoms and signs are headache, nausea, and vomiting, as well as visual field defects and papilledema. MRI imaging can sometimes reveal significant changes, including flattening of the posterior sclera, distension of the perioptic subarachnoid space, and partial empty sella, often correlated to a long lasting elevation of ICP [89]. Clinically, patients typically present with varying combinations of headache, tinnitus, and diplopia [77]. Children with IIH sometimes present with signs that mimic a posterior fossa lesion, including ataxia, nuchal rigidity, facial palsy, or torticollis [89]. Typical symptoms of papilledema include loss of visual acuity and/or transient visual blurring. Papilledema is frequently identified at the time of presentation but could be also observed on routine fundoscopic examination in asymptomatic patients. Ophthalmoplegia can also sometimes occur in patients with IIH, as a result of sixth cranial nerve palsy [89].

While the exact pathophysiology of IIH remains unknown, there have been many proposed theories. Notably, various exogenous and endogenous disorders of the hypothalamic-pituitary-adrenal axis including Addison's disease and Cushing's disease, chronic use of corticosteroids as well as withdrawal from chronic use, adrenal androgen excess and more recently PAL and SAL have been all shown to be potentially associated with the development of IIH [39, 40, 50, 90, 91].

A recent study proposed a theory unifying various neuroendocrine effects on the mineralocorticoid receptor (MR) pathway to explain a possible mechanism for the increased cerebrospinal fluid (CSF) production and ICP in IIH [50, 92]. The MR(s) are abundantly expressed in the choroid plexus epithelial cells (CPEC), which are putatively crucial in the regulation of CSF production [93]. Activation of the MR or its downstream pathways can enhance and stimulate the generation of Na/K ATPase pumps, which can lead to the movement of sodium ions at the CPEC apical membrane into the cerebral ventricle and actively create an osmotic gradient to drive CSF secretion and increase CSF pressure [94, 95]. Based on this perspective, the MR signalling at the CPEC level could therefore be a key pathway in IIH pathophysiology and could explain several reported endocrine-metabolic causes of IIH (see Figure 3), including PAL and SAL, obesity, metabolic syndrome, Cushing syndrome, chronic steroid administration, hypervitaminosis A, recombinant growth hormone (r-GH) therapy, and estro-progestin supplementation [50, 89–91].

Aldosterone, a mineralocorticoid responsible for Na^+^ reabsorption and K^+^, Ca^2+^, and Mg^2+^ excretion in target tissues, including the CPEC, can exert its biological effects on these cells via the MR pathway [50]. An increase in its activity in PAL and SAL disorders may potentially directly affect the ICP in IIH. Support for this perspective includes numerous recent studies demonstrating that in children and adults with PAL or SAL, those treated with spironolactone, an aldosterone receptor antagonist, had resolution of the neurological symptoms and of the ophthalmological manifestations [95, 96]. Additional paediatric cases further strengthened this association of IIH and hyperaldosteronism in which children with various conditions (e.g., metabolic syndrome, SAL due tubular dysfunction) have been successfully treated with spironolactone after a lack of clinical response to the other diuretic treatments (e.g., acetazolamide) [95–97].

This emergent perspective has been proposed as potentially unifying because of the many reported endocrine metabolic associations that may have a common action on the MR pathway, reflecting the possible important involvement of the adrenocortical hormones in the homeostasis of CSF production and pressure [50, 92].

CSF cortisol levels are regulated by 11*β*HSD1, that is abundant the CPEC and converts inactive cortisone to cortisol and acts with high affinity at the MR(s) (similarly to aldosterone) in the CPEC; a pathophysiological link between the enzyme activity and the predisposition to IIH has therefore been suggested [98].

Thus, derangements of this putative adrenal-brain axis in children, through exogenous or endogenous mechanisms, may lead to the development of IIH via this mechanism. Vitamin A has been shown to induce expression of neurosteroids in glial cell lines, which could also theoretically interact with MR(s) [99]. Additionally, human fat, an active endocrine tissue, secretes various cytokines and aldosterone-releasing factors, providing another possible link to elevated ICP in obese patients with IIH (in addition to the link of aldosterone-related predisposition to arterial hypertension, insulin resistance, and metabolic syndrome in the obese population) [50, 100, 101].

Finally, a relationship between IIH and r-GH therapy has been reported numerous times and r-GH is known to be associated with RAS activation and elevated aldosterone levels, especially in the first phases of treatment [102, 103]. Thus, this emerging perspective suggests that the above mentioned associations with IIH may all have a unified action on the MR pathway in the CP, through the adrenal-brain axis, resulting in altered CSF fluid dynamics and elevated ICP (Figure 3) [103, 104].

However, further experimental work should to be performed to confirm these potential perspectives for a complete understanding of the pathophysiology of IIH when related to other reported risk factors (e.g., adrenal insufficiency, steroid withdrawal) and to assess the best etiologically targeted treatment for this increasingly recognised neurological disorder.

## 5. Disorders of the Adrenal Medulla and the Paediatric Brain

The adrenal medulla is located at the centre of the adrenal gland, is surrounded by the adrenal cortex, and consists of secreting cells called “*chromaffin cells*” (or pheochromocytes because they stain brown with chromium salts) that secrete* epinephrine* (adrenaline),* norepinephrine* (noradrenaline), and a small amount of* dopamine* in response to stimulation by* sympathetic pre-ganglionic neurons* [72].

Catecholamine-secreting tumours of the adrenal medulla are called pheochromocytomas, which are very rare tumours in children; they can be solitary or multiple, benign or malignant and are frequently associated with an underlying genetic disease (Figure 4). Those tumours arising in the sympathetic ganglia are called extra-adrenal paragangliomas [72].

Some triggering factors, such as intercurrent illness, hypoglycaemia, and surgical procedures, increase the production of catecholamines from the adrenal medulla with a subsequent impact mainly on the cardiovascular system and onset of manifestations such as increasing heart frequency, elevation of blood pressure, increased myocardial contractibility, and development of cardiac conduction anomalies [72].

Clinical manifestations of pheochromocytomas and paragangliomas are related to catecholamine action on the cardiovascular system, with some other symptoms that include increased (cold) sweating, tremors, weakness, and psychological agitation associated with palpitations [10]. Tumours that affect the adrenal medulla cause increased secretion of norepinephrine and epinephrine. Tumours that secret norepinephrine usually produce severe sustained hypertension, whereas those that secrete primarily epinephrine produce episodic hypertensive crises [72].

Neurologic complications are usually caused by changes in blood pressure and include episodic headaches, and ischemic or haemorrhagic cerebrovascular events have been reported in the paediatric literature [105–107]. Furthermore, it is important to be cognisant of the possibility of posterior reversible encephalopathy syndrome (PRES) in children with pheochromocytoma or paraganglioma presenting with hypertension and cerebrovascular manifestations [108]. PRES is a recently recognised clinical-radiological entity, previously called hypertensive encephalopathy. In fact, arterial hypertension could be regarded as the most well-known risk factor for this condition, and therefore, several children with PRES caused by pheochromocytoma or paraganglioma have been reported in the literature [109–111].

Clinically, children with PRES typically manifest headache, encephalopathy, confusion, visual symptoms, and seizures [108, 110]. Typical MRI changes predominantly involve the white matter of territories supplied by the posterior cerebral circulation (Figure 5), and the radiological abnormalities as well as the clinical manifestations are usually reversible, once the causal factor (e.g., hypertensive crisis) returns to within normal physiological limits.

Correct and timely diagnosis of this condition in children has important therapeutic and prognostic implications because the reversibility of the clinical and radiologic abnormalities is contingent on the prompt control of the blood pressure. Although the pathophysiology of PRES is still unclear, the current most accepted theory is that severe hypertension exceeds the limits of autoregulation, leading to breakthrough brain oedema and the onset of neurological manifestations coupled with correlated radiological findings [110].

Interestingly, some authors postulated that the risk of hypertension-related PRES is higher in the paediatric population compared to the adults due the immaturity of the regulatory mechanisms that protect the brain from damage related to blood pressure elevations [112].

### 5.1. Genetic Disorders with Pheochromocytoma

At least 24% of pheochromocytomas and sympathetic paragangliomas have been estimated to be correlated with familial cancer syndromes and various genetic disorders [51, 52, 113]. Identification of these syndromes and disorders is therefore of prime importance for these children and their relatives.

Multiple endocrine neoplasia type 2 (MEN 2) is a distinct hereditary syndrome that has an autosomal dominant pattern of inheritance and different subtypes (e.g., MEN 2A; MEN 2B), associated with specific mutations in the proto-oncogene* RET* [52, 114, 115].

*Multiple endocrine neoplasia type 2A* (MEN 2A; MIM 171400) is an autosomal dominant disease characterised by parathyroid hyperplasia or adenoma, medullary carcinoma of the thyroid, and bilateral pheochromocytomas [114, 115].

*Multiple endocrine neoplasia type 2B* (MEN 2B; MIM 162300) is also an autosomal dominant disorder and is phenotypically characterised by the combination of pheochromocytomas, mucosal neuromas, and thickening of the optic nerves. Patients with MEN 2 B also develop medullary thyroid carcinoma (100%) and may also have intestinal ganglioneuromatosis. Although medullary thyroid cancer and pheochromocytoma account for most of the morbidity and mortality associated with MEN 2B, the nonendocrine physical findings are important in identifying at-risk individuals early in life [52]. Patients with MEN 2B often have skeletal abnormalities such as talipes equinovarus, pes cavus, dorsal scoliosis, kyphoscoliosis, and lordosis; small joint hyper laxity and chest deformities (e.g., pectus excavatum) are also common clinical findings (Figures 6(a) and 6(b)). Almost 100% of patients with MEN 2B have mucosal neuromas and abnormal dentition (Figures 6(c) and 6(d)) [52].

*Von Hippel-Lindau disease* (VHL; MIM 193300) is an autosomal dominant familial neoplasia syndrome that results from a germline mutation of the* VHL* gene. It is characterised by the presence of paragangliomas, pheochromocytomas, retinal angiomas, cerebellar hemangioblastomas, renal and pancreatic cysts, and renal cell carcinomas [51].

*Neurofibromatosis type 1* (NF1; MIM 162200) is an autosomal dominant disease characterised by café-au-lait spots, axillary/inguinal freckling, iris hamartomas, neurofibromas, optic nerve gliomas, and skeletal abnormalities including sphenoid dysplasia, caused by mutations in the* NF1* gene [116, 117].

Pheochromocytomas are a very rare feature of NF, affecting approximately 0.1% to 6% of all patients, although a study suggested that they may be missed in some NF1 patients [118]. However, NF-1 associated pheochromocytomas occur in adults and very rarely in paediatric patients [119] and almost never in other NF-related phenotypes [120, 121].

*Familial paragangliomas* are a group of autosomal dominant disorders caused by mutations in the genes encoding the succinate dehydrogenase (SDH) mitochondrial complex and are characterised by paragangliomas, usually located in the head and neck [52]. These tumours are usually benign, although approximately 10% of them may undergo malignant transformation, depending on their local invasion and degree of vascularisation. The prognosis depends on the extension of the disease at the time of the diagnosis [114].

## 6. Conclusions

The paediatric nervous system is vulnerable to potential insults during a wide critical period, which extends from the first (embryonic) developmental phases through the entire adolescence and involves tight ontogenic regulatory and feedback activities. These activities are mediated by a number of (intrinsic and external) modulators: any perturbation of these activities/modulators could result in long-term consequences leading to (reversible or nonreversible) impairment of the neurological structure(s) and/or function.

The* adrenal hormones *are among the most sophisticated and important regulatory modulators of the cellular and surrounding environment in the developing (i.e., paediatric) nervous system. Thus, physicians should be aware not only to (the well-known) systemic manifestations but also to the frequent potential neurological and/or psychiatric abnormalities related to a wide array of adrenal diseases and to (acute or chronic) exposure to supra- (or infra-) physiological levels of corticosteroids in children so as to achieve better prevention and timely diagnosis and treatment of these disorders. In the present review we focused on the pathophysiological and clinical implications of glucocorticoid-related, mineralcorticoid-related, and catecholamine-related neurological manifestations and/or paediatric brain damage secondary to* endogenous* (i.e., Cushing syndrome, Addison's disease, congenital adrenal hyperplasia, X-linked adrenoleukodystrophy, autoimmune polyglandular syndrome type 1, congenital adrenal hypoplasia, triple A syndrome, Smith-Lemli-Opitz syndrome, Kearns-Sayre syndrome, hyperaldosteronism, pseudohyperaldosteronism and pseudohypoaldosteronism, genetic and nongenetic tumours of the adrenal cortex or medulla) or* exogenous* (e.g., replacement or acute/chronic corticosteroid therapies) exposure to low or high levels of adrenal hormones.

## Figures and Tables

**Figure 1:** A 5-year-old girl with Cushing Syndrome due to adrenal adenoma that we followed up at our Institution (University of Messina) for sleep disturbances and mood disorders. Note the characteristic facial plethora.

**Figure 2:** Brain MRI. Newborn with classic adrenal congenital hyperplasia, on day 12 after birth, white matter abnormalities that consisted of bilateral small diffuse hyperintensities (white arrow) are depicted on T1-weighted images (a). At 1 yr. of age, bilateral small diffuse hyperintensities are documented (white arrow) on T1-weighted images (b). (Reprinted with permission from [49], Copyright Japanese Society for Pediatric Endocrinology).

**Figure 3:** The putative effects of a wide array of neuroendocrine interactions on CSF secretion in the choroid plexus epithelium. Detailed figure of CP epithelium illustrating the proposed regulation of CSF secretion by several neuroendocrine interactions. Aldosterone can stimulate MR. In nucleus MR can activate mineralocorticoid responsive elements that stimulate synthesis from DNA of Na^+^/K^+^ ATPase pumps. Active sodium secretion by the Na/K ATPase at the apical CP membrane lead to movement of sodium ions into the cerebral ventricle and this creates an osmotic gradient to drive CSF secretion. The enzyme 11*β*HSD1 is highly abundant in the CP, in which its oxidoreductase activity converts inactive cortisone to cortisol, which can activate the MR with similar affinity to aldosterone. All-trans retinoic acid, interacting with DNA, can activate neurosteroidogenesis and* de novo* synthesis of steroids. CPEC = choroid plexus epithelial cells; CSF = cerebrospinal fluid; MR = mineralcorticoid receptor; CSF = cerebrospinal fluid; see [50] (http://www.ncbi.nlm.nih.gov/pubmed/23160227).

**Figure 4:** (a) Bilateral pheochromocytomas (arrows) with rim enhancement in the adrenal glands of a 26-year-old woman with VHL disease; (b) Pheocromocytomas tumor cells are arranged in rounded clusters, separated by endothelial-lined spaces, with have vesicles containing norepinephrine and epinephrine (Reprinted with permission from [51], Copyright Springer Verlag). VHL = Von Hippel − Lindau.

**Figure 5:** FLAIR brain MR images of a 12-year-old girl with sporadic paraganglioma admitted to our Institution with headache and seizures. Unilateral right occipitoparietal lobe vasogenic edema (arrows), typical of PRES, is well depicted after a severe hypertensive crisis. PRES = Posterior reversible encephalopathy syndrome.

**Figure 6:** Clinical Features of MEN2B syndrome. Note (a) the laxity in the first metacarpal joint with complete hyperextension causing no pain; (b) typical chest deformity with pectus excavatum; (c) mucosal neuroma in the anterior tongue; (d) abnormal dentition (Reprinted with permission from [52], Copyright Springer Verlag). MEN2B = Multiple endocrine neoplasia type 2b.
